The article "Forkhead-box C1 attenuates high glucose-induced trophoblast cell injury during gestational diabetes mellitus via activating adenosine monophosphate-activated protein kinase through regulating fibroblast growth factor 19" was retracted in 2024. Reasons: original data or images not available; concerns about the data; concerns about the results or conclusions.

# Forkhead-box C1 attenuates high glucose-induced trophoblast cell injury during gestational diabetes mellitus via activating adenosine monophosphate-activated protein kinase through regulating fibroblast growth factor 19

**DOI:** 10.1080/21655979.2021.2018094

**Published:** 2022-01-04

**Authors:** Shan Cao, Shuxuan Zhang

**Affiliations:** Department of Obstetrics, Xuzhou First People’s Hospital, Xuzhou, China

**Keywords:** FOXC1, trophoblast cell injury, gestational diabetes mellitus, AMPK, FGF19

## Abstract

Gestational diabetes mellitus (GDM) is a complication developed during pregnancy and recover after childbirth. The purpose of this study was to investigate the protective role of FOXC1 during GDM and the underlying mechanism. FOXC1 was downregulated in GDM placental tissues and HG-treated HTR-8/SVneo cells. Overexpression of FOXC1 prevented HG-induced inhibition of cell proliferation, migration and invasion. FOXC1 suppressed HG-induced cell apoptosis in HTR-8/SVneo cells. The apoptosis-related proteins: cleaved caspase-3, cleaved caspase-9 and BAX, were also downregulated by FOXC1 overexpression. FOXC1 increased glucose uptake and improved insulin sensitivity. The expression of FOXC1 was positively correlated with FGF19 expression. FOXC1 regulated the expression of FGF19 and phosphorylation of AMPK. Inhibition of FGF19 attenuated the biological functions of FOXC1 through inactivation of AMPK. In conclusion, this study demonstrates that FOXC1 attenuates HG-induced trophoblast cell injury through upregulating FGF19 to activate the AMPK signaling pathway during GDM, suggesting that FOXC1 is a potential therapeutic target for drug discovery in the future.

## Introduction

Gestational diabetes mellitus (GDM) is a metabolic disorder developed during pregnancy and recover after childbirth [1]. So far, there is no consensus in term of the diagnostic criteria for GDM. As recommended by the International Association of Diabetes and Pregnancy Study Group (IADPSG), GDM is characterized by fasting plasma glucose (FPG) ≥ 92 mg/dL or glucose tolerance test (OGTT) 75 g within 2 h when FPG < 92 mg/dL at the first prenatal visit [1]. According to estimates from International Diabetes Federation (IDF) in 2017, ~14% of pregnant women are diagnosed with GDM [2]. Almost 90% of GDM cases are diagnosed in low- and middle-income countries, and the occurrence of GDM is associated with obesity, race, westernized diet, and excessive gestational weight gain [2].

The pathophysiology of GDM is complex and multi-organ related, including pancreatic β cell dysfunction, adipose tissue, chronic insulin resistance, liver and placenta [3]. Adenosine monophosphate (AMP)-activated protein kinase (AMPK) is an essential serine/threonine kinase that maintains the normal function of placental tissues during pregnancy [4]. It is also an intracellular energy sensor that improves insulin sensitivity through enhancing glucose uptake in metabolic syndrome [5]. During GDM, AMPK activity is inhibited, resulting in the disruption of glucose metabolism and energy homeostasis, impairment of insulin sensitivity and nutrient transportation [6]. Therefore, activation of AMPK might prevent the occurrence of GDM.

FOXC1 is a transcription factor, which belongs to human forkhead-box (FOX) gene family [7], and takes part in cell growth, mobility, differentiation and apoptosis in various cancers [8]. Besides cancer, *FOXC1* transcripts have also been also detected in the embryonic tissues [9]. *FOXC1*-knockout pregnant mice deliver dead fetus with many organ defects, including dysfunction of central nervous system, eye defects, and skeletal abnormalities [9]. Furthermore, FOXC1 was also reported to affect ovarian function [10]. Migration of primordial germ cells is impaired in *FOXC1* mutant mice, resulting in insufficient movement to reach the gonadal anlage [11]. Thus, in the current study, we hypothesized that FOXC1 plays a protective role during GDM. We aimed to investigate the role of FOXC1 in GDM and the underlying mechanism to provide a better understanding of GDM and identify potential management targets for GDM.

## Materials and methods

### Human sample collection

Placental tissues (1 cm at the central part) were collected immediately after birth from 13 normal pregnant women (NP) and 9 pregnant women with GDM (Table 1) at Xuzhou First People’s Hospital. Each placental tissue was divided into two: half of them was submerged in the Carnoy Fixation Solution (GefanBio, China), and another half was stored at −80°C. Written informed consent were collected from all patients for sample analysis and data publication. This study complied with the Declaration of Helsinki [12] and the protocol was approved by the Ethics Committee of Xuzhou First People’s Hospital. The diagnosis of GDM was made in accordance with the Guideline No. 393-Diabetes in Pregnancy: fasting plasma glucose ≥ 5.1 mmol/L, 1-hour plasma glucose ≥ 10.0 mmol/L and/or 2-hour plasma glucose ≥ 8.5 mmol/L using a standardized 2-hour 75-g oral glucose tolerance test [13].

**Table 1.** Clinical information

Subjects	NP (N = 13)	GDM (N = 9)	P value
Age (Y)	29.38 ± 2.16	30.11 ± 2.28	
Gestational week (W)	39.07 ± 0.83	39.44 ± 0.83	
Pre-maternal BMI (kg/m^2^)	21.33 ± 0.46	21.91 ± 0.35	P = 0.0067**
Maternal weight gain(kg)	12.97 ± 0.50	13.3 ± 0.53	
OGTT FPG (mmol/L)	4.49 ± 0.07	5.08 ± 0.0.19	P < 0.001***
OGTT 1hPG (mmol/L)	8.47 ± 0.23	10.29 ± 0.28	P < 0.001***
OGTT 2hPG (mmol/L)	7.42 ± 0.15	8.32 ± 0.24	P < 0.001***
HDL (mmol/L)	1.73 ± 0.41	1.88 ± 0.59	
LDL (mmol/L)	2.87 ± 0.47	3.29 ± 0.76	
Fetal birth weight (g)	3288 ± 76.69	3606 ± 126.8	P < 0.001***
Placental weight (g)	492.1 ± 64.23	529.8 ± 63.5	

*p < 0.05.

## Cell culture and transfection

Human trophoblast cell line, HTR-8/SVneo, was obtained from Wuhan Procell Life Science & Technology Co., Ltd (Procell, China). RPMI-1640 medium (VivaCell, China) was supplemented with 10% fetal bovine serum (FBS, VivaCell) and 1% penicillin-streptomycin solution (100×, Solarbio, China). HTR-8/SVneo cells were cultured with supplemented RPMI-1640 medium at 37°C with 5% CO_2_ in a humid incubator.

Normal glucose referred to 5 mM glucose in the culture medium, whereas high-glucose (HG) treatment in this study referred to adding extra 25 mM glucose (Sigma-Aldrich) into the normal culture medium. For each experiment, HTR-8/SVneo cells were seeded into 6-well plates at a density of 1 × 10^6^ cell/well and cultured to 80% confluency before treatment.

The coding sequence of *FOXC1* (Sigma-Aldrich, USA) or its negative control (NC) was cloned into pGL3 vectors (YouBio, China) to generate pGL3-FOXC1 and pGL3-NC plasmids, respectively. Small interfering RNA (siRNA) targeting fibroblast growth factor 19 (FGF19) (siFGF19) was purchased from Suzhou Biosyn Technology Co., Ltd (Biosyn, China). Cell transfection was performed using the LipoGene™ 2000 PLus Transfection Reagent (Yuhengbio, China) following the manufacturer’s protocols.

## Flow cytometry

Cell apoptosis was determined using flow cytometry [14]. After treatment, cells were collected and stained using the Annexin V-FITC/PI Apoptosis Detection Kit (Qcbio) for 15 min at room temperature in dark. 20,000 cells were collected for analysis using FACS Calibur flow cytometer (BD, USA).

## CCK-8 and EDU assays

Cell viability was examined using the Cell Counting Kit-8 (CCK-8 kit, Beyotime, China) [15] and the data of CCK-8 assays was read using a microplate reader (Hengmei, China). Cell proliferation was detected using the C and BeyoClick™ EdU Cell Proliferation Kit with Alexa Fluor 555 (Beyotime) according to manufacturer’s instructions. Results from the EDU assays were recorded using a flow cytometer.

## Transwell assay

Cell migration and invasion were assessed using Transwell assay [16]. To detect cell migration, treated HTR-8/SVneo cells were resuspended in FBS-free medium and seeded into the upper chamber of a 24-well insert (8-μm pore size; Corning, USA). FBS-supplemented medium was added to the lower chamber. After incubation at 37°C for 48 h, cells were fixed with 4% paraformaldehyde (Solarbio, China) for 30 min at 4°C and stained with 1% crystal violet solution (Solarbio). Migrated cells were imaged and the number of migrated cells was counted using an inverted microscope (Leica, Germany). For the detection of cell invasion, the upper chamber of a 24-well insert was precoated with Matrigel (Solarbio) and the experiment was performed using the same protocols as cell migration assay.

## Measurement of glucose uptake

Glucose uptake was measured using the Glucose Uptake Assay Kit according to manufacturer’s protocols. The results were read and analyzed using a microplate reader.

## Quantitative real-time polymerase chain reaction (qRT-PCR)

qRT-PCR was carried out as previously described [17]. Total RNA was extracted using TRIzol RNA Isolation Reagent (Thermo Fisher, USA). Reverse transcription was performed using the RevertAid RT Reverse Transcription Kit (Thermo Fisher) and amplification was conducted using RNA UltraSense™ One-Step Quantitative RT-PCR System (Thermo Fisher). Relative mRNA expression was calculated using 2^−ΔΔCT^ method. *GAPDH* was used as the reference gene for data analysis. Primer sequences (RiboBio) used in this study are as follows: *FOXC1* forward 5ʹ- GGCGAGCAGAGCTACTACC-3ʹ and reverse 5ʹ-TGCGAGTACACGCTCATGG-3ʹ; *FGF19* forward 5ʹ-CGGAGGAAGACTGTGCTTTCG-3ʹ and reverse 5ʹ-CTCGGATCGGTACACATTGTAG-3ʹ; and *GAPDH* forward 5ʹ-TGTGGGCATCAATGGATTTGG-3ʹ and reverse 5ʹ-ACACCATGTATTCCGGGTCAAT-3ʹ.

## Western blotting

Western blotting was performed as previously described [18]. Protein isolation was performed using M-PER™ Mammalian Protein Extraction Reagent (Thermo Fisher). 5 μg of total protein was loaded into 7.5% polyacrylamide gel and separated by electrophoresis. Proteins were then transferred onto PVDF membranes (Merck KGaA, Germany). Membranes were incubated with StartingBlock™ (PBS) Blocking Buffer (Thermo Fisher) for 1 h at room temperature and then probed with primary antibodies at 4°C overnight followed by incubation with secondary antibodies for 2 h at room temperature the next day. Protein bands were then visualized using the Efficient chemiluminescence kit (Proandy, China). Primary antibodies (Cell signaling, USA) used in this study are as follows: FOXC1 (#8758, 1:500 dilution), cleaved caspase-3 (#9664, 1:800 dilution), cleaved caspase-9 (#9505, 1:1000 dilution), BAX (#2774, 1:500 dilution), BCL-2 (#1571, 1:500 dilution), GLUT-4 (#2231, 1:500 dilution), INSR-B (#3020, 1:2000 dilution), IRS1 (#2382, 1:2000 dilution), FGF19 (#83,348, 1:1000 dilution), p-AMPK (#2535, 1:2000 dilution), AMPK (#5831, 1:1000 dilution), and β-actin (#3700, 1:5000 dilution).

## Immunohistochemistry (IHC)

Immunohistochemistry was performed as previously described [19]. Fixed placental tissues were embedded in paraffin wax and then cut into 5 µm sections. Xylene was used to deparaffinize the wax section and graded ethanol was used to dehydrate the samples. Epitope retrieval was induced by boiling the sections for 15 min using 10% SignalStain® EDTA Unmasking Solution (Cell Signaling). Sections were blocked using CytoVista™ Blocking Buffer Thermo Fisher) and probed with FoxC1 Rabbit mAb (Cell Signaling). After that, sections were incubated with anti-Rabbit IgG for 2 h at room temperature, followed by incubation with streptavidin-conjugated horseradish peroxidase. Next, sections were submerged in peroxidase substrate, diaminobenzidine (DAB). Images were taken using an inverted microscope.

## Statistical analysis

Statistical analysis was conducted using SPSS 21.0 (SPSS, USA). All data are presented as mean ± SEM. Statistical difference was performed using unpaired student *t*-test (two groups) and one-way ANOVA (multiple groups). All experiment was repeated three times. The correlation between *FOXC1* and *FGF19* mRNA expression was performed using Spearman’s rank-order correlation coefficients. *p* value less than 0.05 was defined as statistical significant.

## Results

In this study, we hypothesized that FOXC1 confers a protective effect during GDM. Thus, we sought to determine the effects of FOXC1 on cell survival and growth in trophoblast cell lines and identify signaling pathway(s) that mediates the protective effects of FOXC1 during GDM.

## FOXC1 is downregulated in GDM placental tissues and HG-treated HTR-8/SVneo cells

The mRNA expression of *FOXC1* was downregulated in GDM placental tissues compared to normal tissues (Figure 1(a)). Consistently, the protein level of FOXC1 was also found to be reduced in GDM placental tissues compared to normal tissues, which was confirmed using Western blotting and IHC (Figure 1(b,c)). Furthermore, FOXC1 was downregulated in HG-treated HTR-8/SVneo cells at both mRNA and protein levels (Figure 1(d,e)). These data demonstrate that FOXC1 is downregulated during GDM.

**Figure 1.** FOXC1 is downregulated in GDM placental tissues and HG-treated HTR-8/SVneo cells. (a) *FOXC1* mRNA is downregulated in GDM placental tissues; (b) Western blot images show that FOXC1 protein is downregulated in GDM placental tissues; (c) IHC images show that FOXC1 protein is downregulated in GDM placental tissues; (d) *FOXC1* mRNA is downregulated in HG-treated HTR-8/SVneo cells; (e) FOXC1 protein is downregulated in HG-treated HTR-8/SVneo cells. **p < 0.01 versus (vs) NP or Control; ***p < 0.005 vs NP or Control. GDM: Gestational diabetes mellitus (n = 9); NP: Normal pregnant women (n = 13); HG: High glucose. FOXC1: forkhead-box C1; IHC: Immunohistochemistry; HG: high glucose.

## FOXC1 promotes cell growth and prevents cell apoptosis in HG-treated HTR-8/SVneo cells

FOXC1 plasmid overexpressed FOXC1 and prevented the reduction of FOXC1 protein induced by HG in HTR-8/SVneo cells (Figure 2(a)). Cell viability and proliferation were increased by FOXC1 overexpression and decreased by HG treatment (Figure 2(b,c)). FOXC1 overexpression reversed HG-induced reduction in cell viability and cell proliferation in HTR-8/SVneo cells (Figure 2(b,c)). Furthermore, cell apoptosis was reduced by FOXC1 plasmid and induced by HG treatment (Figure 2(d)). Overexpression of FOXC1 was able to inhibit HG-induced cell apoptosis (Figure 2(d)). In addition, downregulation of cleaved caspase-3, cleaved caspase-9, BAX, and upregulation of BCL-2 were observed in HG-treated HTR-8/SVneo cells, whereas FOXC1 overexpression suppressed HG-mediated expression changes in these proteins in HTR-8/SVneo cells (Figure 2(e)). Overexpression of FOXC1 also reversed HG-mediated reduction in cell migration in HTR-8/SVneo cells (Figure 3). These results indicate that FOXC1 overexpression blocks HG-mediated inhibition in cell growth and induction in cell apoptosis in HG-treated HTR-8/SVneo cells.

**Figure 2.** FOXC1 promotes cell proliferation and prevents cell apoptosis in HG-treated HTR-8/SVneo cells. (a) Overexpression of FOXC1 reverses HG-induced downregulation of FOXC1; (b) Overexpression of FOXC1 reverses HG-induced reduction in cell viability; (c) Overexpression of FOXC1 reverses HG-induced inhibition of cell proliferation; (d) Overexpression of FOXC1 inhibits HG-induced cell apoptosis; (e) Overexpression of FOXC1 reverses HG-induced dysregulated expression of cleaved caspase-3, cleaved caspase-9, BAX and BCL-2. *p < 0.05; **p < 0.01; ***p < 0.005. FOXC1: pGL3 vector containing the coding sequence of FOXC1; NC: negative control of FOXC1.

**Figure 3.** FOXC1 promotes cell migration and invasion in HG-treated HTR-8/SVneo cells. Overexpression of FOXC1 reverses HG-induced inhibition of cell migration and invasion. **p < 0.01; ***p < 0.005.

## FOXC1 enhances cell sensitivity to insulin in HG-treated HTR-8/SVneo cells

FOXC1 overexpression increased the expression of GLUT4, INSR-B and IRS1 in HG-treated HTR-8/SVneo cells (Figure 4(a)). HG-induced reduction in GLUT4, INSR-B and IRS1 was reversed by overexpressing FOXC1 (Figure 4(a)). In addition, glucose uptake was also increased in HTR-8/SVneo cells transfected with FOXC1 plasmid and decreased in cells treated with HG (Figure 4(b)). Upregulation of FOXC1 increased insulin (100 nM)-induced glucose uptake (Figure 4(b)). Altogether, these data indicate that FOXC1 overexpression enhances cell sensitivity to insulin in HG-treated HTR-8/SVneo cells.

**Figure 4.** FOXC1 enhances cell sensitivity to insulin in HG-treated HTR-8/SVneo cells. (a) Overexpression of FOXC1 reverses HG-induced downregulation of GLUT-4, INSR-B and IRS1; (b) Overexpression of FOXC1 enhances insulin-induced glucose uptake. *p < 0.05; **p < 0.01; ***p < 0.005. GLUT-4: glucose transporter 4; INSR-B: insulin receptor B; IRS1: insulin receptor substrate 1.

## FOXC1 activates the AMPK signaling pathway via FGF19

Next, we found that the transcript level of *FGF19* was lower in GDM placental tissues compared to normal control (Figure 5(a)). Importantly, a positive correlation was observed between the mRNA expression of *FOXC1* and *FGF19* (Figure 5(b)). Transfection of FOXC1 plasmid led to an upregulation of FGF19 and prevented HG-mediated reduction in FGF19 protein in HTR-8/SVneo cells (Figure 5(c)). Phosphorylation of AMPK was also induced by FOXC1 overexpression and inhibited by HG treatment (Figure 5(c)). Furthermore, FOXC1 overexpression was able to reverse HG-mediated inhibition in AMPK phosphorylation (Figure 5(c)). FGF19 silencing by siFGF19 attenuated FOXC1-induced upregulation in FGF19 and phosphorylation of AMPK (Figure 5(d)). Thus, these data suggest that FOXC1 activates the AMPK signaling pathway via upregulation of FGF19.

**Figure 5.** FOXC1 activates the AMPK pathway via FGF19. (a) *FGF19* mRNA is downregulated in GDM placental tissues; (b) The expression of *FOXC1* mRNA is positively correlated with the expression of *FGF1*9 mRNA; (c) Inhibition of FGF19 expression and AMPK phosphorylation induced by HG is reversed by upregulation of FOXC1; (d) FGF19 silencing reverses FOXC1-induced upregulation of FGF19 and phosphorylated AMPK. *p < 0.05; **p < 0.01; ***p < 0.005. FGF19: fibroblast growth factor 19; AMPK: adenosine monophosphate-activated protein kinase; p-AMPK: phosphorylation of AMPK.

## FGF19 silencing contributes to HG-induced injury in HTR-8/SVneo cells

FGF19 silencing inhibited FOXC1-induced cell proliferation in HG-treated HTR-8/SVneo cells (Figure 6(a)). Cell apoptosis induced by HG treatment was inhibited by overexpression of FOXC1 and this inhibition was attenuated by FGF19 knockdown (Figure 6(b)). Cell migration and invasion were increased by FOXC1 overexpression, but this was blocked when FGF19 was silenced (Figure 6(c)). Moreover, the expression of GLUT4, INSR-B and IRS1 was increased by FOXC1 overexpression and this was reversed by silencing FGF19 (Figure 6(d)). Altogether, these findings demonstrate that downregulation of FGF19 contributes to HG-induced injury in HTR-8/SVneo cells.

**Figure 6.** FGF19 silencing contributes to HG-induced injury in HTR-8/SVneo cells. (a) FGF19 silencing prevents FOXC1-induced cell proliferation; (b) FGF19 knockdown reverses FOXC1-induced inhibition of cell apoptosis; (c) Downregulation of FGF19 prevents FOXC1-induced cell migration and invasion; (d) FGF19 silencing reverses FOXC1-induced upregulation of GLUT-4, INSR-B, IRS1. *p < 0.05; **p < 0.01; ***p < 0.005.

## Discussion

Although GDM recovers after delivery, the affected women are still under high risk of developing diabetes over time [20]. GDM offspring is also affected by GDM with an increased risk of developing insulin resistance, neurodevelopmental impairments and disorder of glucose metabolism [20]. Thus, understanding the mechanism of GDM is important to facilitate the prevention and management of GDM. In the present study, FOXC1 was found to be downregulated in GDM placental tissues and HG-treated HTR-8/SVneo cells. FOXC1 overexpression promoted cell growth and mobility, increased glucose uptake and improved insulin sensitivity. FGF19 silencing inhibited the effects of FOXC1 in GDM and reduced the activity of AMPK. These data demonstrate that the beneficial effects of FOXC1 are mediated by activation of AMPK through upregulation of FGF19.

Placental lesions induced by cell death are related to many fetal growth restrictions, including preeclampsia, metabolic disorders, and immune dysfunctions [21,22]. Therefore, reduced cell viability and mobility affects placental nutrient transport [22]. In this study, FOXC1 overexpression was found to inhibit apoptosis, increase cell viability and mobility in HG-treated HTR-8/SVneo cells, implying the beneficial effects of FOXC1 on placental cell survival, which is consistent with previous finding that FOXC1 promotes cell proliferation and migration [23]. Insulin has been shown to play a key role in regulating DHA transfer, amino acid transport, and glucose transport in trophoblasts [24–26]. Data from this study have shown that HG reduced glucose uptake and impaired insulin sensitivity in trophoblasts and this was reversed by FOXC1 overexpression, suggesting that FOXC1 plays a key role in the normal functions of placenta to maintain nutrient supply during GDM. This is the first time that the protective effects of FOXC1 in GDM were reported. Activation of AMPK is known to increase glucose uptake through enhancing insulin-stimulated GLUT4 expression [27]. Our findings have demonstrated that the expression of GLUT4 and phosphorylation of AMPK were positively regulated by FOXC1. These indicate that the protective effects of FOXC1 on cell survival and glucose uptake are mediated by AMPK phosphorylation, implying that AMPK is a potential therapeutic target for GDM.

Fibroblast growth factor 19 (FGF19) is a crucial protein that regulates glucose metabolism and maintains energy homeostasis [28]. In this study, FGF19 silencing reduced glucose uptake and impaired insulin resistance in HG-treated HTR-8/SVneo cells, resulting in the disruption of energy homeostasis during GDM. Moreover, inhibition of FGF19 promoted cell death and reduced cell growth, indicating that FGF19 prevented trophoblast cell injury during GDM. FOXC1 has been reported to directly activate the transcription of FGF19 to upregulate FGF19 expression in corneal cells and zebrafish embryos [29]. In this study, FOXC1 was found to upregulate the expression of FGF19. Furthermore, FGF19 knockdown attenuated the effects of FOXC1 on HG-treated HTR-8/SVneo cells, demonstrating that the protective effects of FOXC1 on trophoblast cells were mediated by regulating FGF19 expression during GDM. Several studies have revealed that FGF19 could promote the phosphorylation of AMPK [29–31]. In agreement with previous findings, the data from this study have shown that FGF19 silencing inhibited the phosphorylation of AMPK. Taken together, FGF19 mediates the protective effects of FOXC1 through upregulating phosphorylated AMPK during GDM, providing a new insight into GDM and suggests a potential new target for drug discovery in the future.

## Conclusion

In conclusion, the findings from this study indicate that inhibition of FOXC1 expression contributes to cell apoptosis and cell death during GDM. The expression of FGF19 expression is positively correlated with FOXC1 expression. Inhibition of FGF19 suppresses the beneficial effects of FOXC1 on GDM and reduces AMPK activity. Thus, the beneficial effects of FOXC1 on trophoblast cell survival are mediated by activation of AMPK through upregulation of FGF19. This study provides a better understanding of the pathophysiological mechanism underlying GDM and facilitates the prevention and management of GDM in the future.

## Data Availability

All data generated or analyzed during this study are included in this published article.

## Highlight

- FOXC1 was downregulated in GDM placental tissues and HG-treated HTR-8/SVneo cells.
- FOXC1 promoted cell growth and prevented cell apoptosis in HG-treated HTR-8/SVneo cells.
- FOXC1 enhanced cell sensitivity to insulin in HG-treated HTR-8/SVneo cells.
